The article "Identification and Potential Mechanisms of a 7-MicroRNA Signature That Predicts Prognosis in Patients with Lower-Grade Glioma" was retracted in 2023. Reasons: signs of a paper mill; compromised peer review; unreliable results or conclusions.

# Identification and Potential Mechanisms of a 7-MicroRNA Signature That Predicts Prognosis in Patients with Lower-Grade Glioma

**DOI:** 10.1155/2021/3251891

**Published:** 2021-11-20

**Authors:** Zhizheng Liu, Hongliang Meng, Miaoxian Fang, Wenlong Guo

**Affiliations:** ^1^Department of Neurosurgery, The First Affiliated Hospital of Nanchang University, Nanchang, China; ^2^Department of Neurosurgery, Guangdong Provincial People's Hospital, Guangdong Academy of Medical Sciences, Guangzhou, China; ^3^Department of Neurosurgery, Gan Zhou People's Hospital, Gan Zhou, China; ^4^Department of Intensive Care Unit of Cardiac Surgery, Guangdong Provincial People's Hospital, Guangdong Academy of Medical Sciences, Guangdong Cardiovascular Institute, Guangzhou, China

## Abstract

**Background:**

Lower-grade glioma is an intracranial cancer that may develop into glioblastoma with high mortality. The main objective of our study is to develop microRNA for LGG patients which will provide novel prognostic biomarkers along with therapeutic targets.

**Methods:**

Clinicopathological data of LGG patients and their RNA expression profile were downloaded through The Cancer Genome Atlas Relevant expression profiles of RNA, and clinicopathological data of the LGG patients had been extracted from the database of “The Cancer Genome Atlas.” Differential expression analysis had been conducted for identification of the differentially expressed microRNAs as well as mRNAs in LGG samples and normal ones. ROC curves and K–M plots were plotted to confirm performance and for predictive accuracy. For the confirmation of microRNAs as an independent prognostic factor, an independent prognosis analysis was conducted. Moreover, target differentially expressed genes of these identified prognostic microRNAs that were extracted and protein-protein interaction networks were developed. Moreover, the biological functions of signature were determined through Genome Ontology analysis, genome pathway analysis, and Kyoto Encyclopedia of Genes.

**Results:**

7-microRNA signature was identified that has the ability of categorization of individuals with LGG into high- and low-risk groups on the basis of significant difference in survival during training and testing cohorts (*P* < 0.001). The 7-microRNA signature had appeared to be robust in predictive accuracy (all AUC> 0.65). It was also approved with multivariate Cox regression along with some traditional clinical practices that we can use 7-microRNA signature for therapeutic purposes as a self-regulating predictive OS factor (*P* < 0.001). KEGG and Gene Ontology (GO) analyses reported that 7-microRNAs had mainly developed in important pathways related with glioma, e.g., the “cAMP signaling pathway,” “glutamatergic synapses,” and “calcium signaling pathway”.

The article "Identification and Potential Mechanisms of a 7-MicroRNA Signature That Predicts Prognosis in Patients with Lower-Grade Glioma" was retracted in 2023. Reasons: signs of a paper mill; compromised peer review; unreliable results or conclusions.

**Conclusion:**

A newly discovered 7-microRNA signature could be a potential target for the diagnosis and treatment for LGG patients.

## 1. Introduction

Gliomas constitute approximately 70% of all primary malignant brain tumors, which are characterized by no clear boundary, diffuse infiltration, and high invasion [1]. The classification by the WHO of gliomas into four different grades was based on histology and molecular parameters [2]. Most of the lower-grade gliomas (LGG) that grow diffusely in the cerebral hemispheres include grade-II and grade-III gliomas [3]. It is difficult to have complete resection due to the highly infiltrative nature of the tumor cells [4]. It has been observed that shortly after surgery, the patient may suffer progression of recurrence of tumor that may be caused by already existing tumor cells. 70% of LGG develop into glioblastomas inevitably which have overall survival less than 10 years [5]. As compared to glioblastoma, the LGG clinical indicators and the therapeutic targets are very few in number. Therefore, the determination of novel prognostic biomarkers as a therapeutic agent for patients with LGG is imperative.

MicroRNAs are a group of short-chain RNAs that lack protein-coding ability. With the increasing understanding of microRNAs, researchers found that microRNAs could regulate the development of cancers through mediating mRNA expression. MicroRNAs have been demonstrated as promising targets for therapy and biomarkers for prognosis of different types of cancers including hepatocellular carcinoma, glioblastoma, and breast cancer [6–8]. Moreover, it has been shown through evidence that microRNAs are associated with the invasion, proliferation, and also the migration of LGG [9, 10].Thus, microRNA may also act as targets and biomarkers in LGG. However, there are few studies reporting that the microRNAs can diagnose LGG in patients by identifying its individual outcomes.

The current study determined the development of a 7-microRNA signature in predicting LGG patient's survival chances utilizing “The Cancer Genome Atlas (TCGA) database.” Besides, the extensive mechanism of the 7-microRNA signature as well as its biological functions were find out using KEGG enrichment analysis and Gene Ontology (GO). This 7-microRNA signature may not only be helpful in the prediction of prognosis of specific patients with LGG but also may determine more pathways of LGG development.

## 2. Materials and Methods

### 2.1. Collection of Data

We downloaded microRNA and mRNA expression profiles for normal and LGG tissues by using the database of TCGA (http://cancergenome.nih.gov/, https://xenabrowser.net/datapages/). Related pathological data from the database of TCGA clinical profiles were also downloaded. Data with missing information were removed. Finally, 477 clinical data of LGG samples were included. These 477 samples were divided randomly into two cohorts according to computer-generated allocation numbers, namely, training and testing cohorts. The approval of institutional ethics was not required as the data were publicly derived using TGGA.

The article "Identification and Potential Mechanisms of a 7-MicroRNA Signature That Predicts Prognosis in Patients with Lower-Grade Glioma" was retracted in 2023. Reasons: signs of a paper mill; compromised peer review; unreliable results or conclusions.

### 2.2. Screening for DEmicroRNAs and DEmRNAs

We used the “edgeR” package (https://cran.r-project.org/) [11] for screening of differentially expressed microRNAs (DEmicroRNAs) in normal tissues and differentially expressed microRNAs (DEmicroRNAs) in LGG tissues. We defined DEmicroRNAs and DEmRNAs with a |log2 (fold change)| ≥1 and false discovery rate (FDR) < 0.05.

### 2.3. Establishment of a Risk Assessment Model

A “survival” package was utilized for the conductance of COX analysis. The DEmicroRNAs were determined from the training cohort by applying univariate and multivariate COX regression coefficients with a *P* value < 0.05. The COX regression analysis was applied for estimation and calculation of microRNAs regression coefficients. So, the development of a microRNA-based risk model was made through independent prognostic DEmicroRNAs. The microRNA-based risk score = sum of regression coefficients x microRNAs expression level. The median risk score was estimated in the training cohort. The categorization of the samples was completed on basis of median risk score that separated the high-risk group from the low-risk group as cutoff value.

### 2.4. Validation of the Prognostic Model

The dispersion of survival status and its rate among these risk groups were visualized using the “survival” package. An assessment of survival difference between both groups on the basis of the testing, training, and entire cohort was made using the Kaplan–Meier curve as well as the log-rank test. The calculations of predictive accuracy of the microRNA signature were obtained from the range under the ROC curve (AUC). Furthermore, the comparison of OS among the low- and high-risk expression group in the risk assessment model was performed through Kaplan–Meier survival analysis [12]. For investigation of effects on independent potential prognostic factors, e.g., age, gender, grade, and risk score, COX hazard regression analyses of the univariate and multivariate types were applied.

### 2.5. Construction of a Coexpression Network

The miRTarBase, miRDB, and TargetScan databases were applied for confirmation of the target DEmRNAs of prognostic microRNAs [13–15]. We preserved target DEmRNAs that were determined through two databases. The selected prognostic microRNAs and the target DEmRNAs were chosen to develop the microRNA-target gene network by utilizing Cytoscape software (version 3.8.0) [16].

The article "Identification and Potential Mechanisms of a 7-MicroRNA Signature That Predicts Prognosis in Patients with Lower-Grade Glioma" was retracted in 2023. Reasons: signs of a paper mill; compromised peer review; unreliable results or conclusions.

### 2.6. Functional Analysis

Functional association of the target genes was found out by uploading the data of these genes on the STRING database [17]. The interaction was significant with combined score >0.4. The top 20 closely interrelated genes were observed utilizing Cytoscape software (version 3.8.0). Thus, all of the target genes in *R* language were exposed to the clusterProfiler package [18] for exploring their novel pathways and potential functions through enriched examination of Gene Ontology (GO) [19] and Kyoto Encyclopedia of Genes and Genomes (KEGG) [20]. Then, KEGG analysis or GO term was measured significant at *P* value <0.05.

### 2.7. Dispersion of the Expression of Diagnostic microRNAs and Risk Score in Different Grades of Glioma

To find the interaction among the risk model and tumor grade, we performed Student's *t*-test to compare the risk score level and expression of different microRNAs in grade-II and grade-III glioma within the TGCA database.

## 3. Results

### 3.1. Identification and Screening of Differentially Expressed microRNAs and mRNAs

After edgeR filtering log2-fold change ([log2FC] ≥ 1) and false discovery rate (FDR) < 0.05 among LGG samples and adjacent normal tissues, we screened an overall 266 of differentially expressed microRNAs and 5449 of differentially expressed mRNAs in our study. The distribution of differentially expressed microRNAs and mRNAs is exhibited through Figure 1. Overall data of 477 individuals of glioma disease had been extracted from database of “The Cancer Genome Atlas.” All of the selected patients were independently categorized as training and testing cohorts.  Table 1 shows baseline features of the testing and training cohorts.

Mainly, the 7 independent microRNAs having an association with the glioma patient's survival were determined by applying analysis through the multivariate COX regression in the training cohort with *P* < 0.05 (Table 2). A predictive model was developed by using the following calculation: risk score = (−0.398 × expression value of hsa-miR-181a-2-3p) + (−0.361 × expression value of hsa-miR-3200-3p) + (0.328 × expression value of hsa-miR-92b-5p) + (0.118 ×expression value of hsa-miR-10b-5p) + (0.287 × expression value of hsa-miR-221-3p) + (−0.225 ×  hsa-miR-548ba) + (−0.321 × hsa-miR-153-5p). In this model, hsa-miR-92b-5p, hsa-miR-10b-5p, and hsa-miR-153-5p were positive coefficients, and negative coefficients include hsa-miR-181a-2-3p, hsa-miR-3200-3p, hsa-miR-548ba, and hsa-miR-153-5p (Table 2). This predicted that LGG patients with high expression profiles for hsa-miR-92b-5p, hsa-miR-10b-5p, and hsa-miR-153-5p had better survival, while those with high expression of hsa-miR-181a-2-3p, hsa-miR-3200-3p, hsa-miR-548ba, and hsa-miR-153-5p had poor survival.

The article "Identification and Potential Mechanisms of a 7-MicroRNA Signature That Predicts Prognosis in Patients with Lower-Grade Glioma" was retracted in 2023. Reasons: signs of a paper mill; compromised peer review; unreliable results or conclusions.

### 3.2. Verifying the Predictive Performance of the 7-microRNA Signature in Different Cohorts

The basis of classification was the training cohort, threshold, entire cohort, and testing cohort with median risk score which divides those samples into groups with high and low risk.  Figure 2(a) exhibits the dispersion among the survival status and time of survival. Visual inspection revealed that LGG individuals with higher risk score have lower “overall survival” rate than individuals of the low-risk group in all cohorts. Kaplan–Meier analysis in the training cohort identified that the low-risk group tends to have more survival time rather than the high-risk group (*P* value < 0.001) (Figure 2(b)). The AUC for the ROC curves in the training cohort showed sensitivity and specificity of the risk model (AUC = 0.914) (Figure 2(c)). Additionally, the analysis of LGG patients in the testing (*P* value < 0.001, AUC = 0.887) and entire cohorts (*P* value < 0.001, AUC = 0.906) also confirmed the predictive power of the 7-microRNA biomarkers. These results exhibited the firm diagnostic value of the 7-microRNA risk score model. For the 3 risky microRNAs, the member in the low-risk category tends to exhibit higher survival rate as compared to other groups (*P* < 0.05) as exhibited in Figure 3. For the 4 protective microRNAs, the member in the low expression group had probably lower OS value than those in the higher expression group.

### 3.3. The Independence of the 7-microRNA Signature for Survival Prediction

Univariate and multivariate Cox regressions were made for the assessment of the self-regulating prognostic value of the 7-microRNA signature along with the associated clinical factors. These clinical factors included age (≥42 vs. <42), gender (female vs. male), and tumor grade (III vs. II). The outcomes of univariate COX regression analysis, except for gender (HR = 1.063, 95% CI 0.742–1.522, *P* = 0.739), risk score model (HR = 1.135, 95% CI 1.109–1.162, *P* < 0.00V01), age (HR = 1.058, 95% CI 1.043–1.074, *P* < 0.0001), and tumor grade (HR = 3.313, 95% CI 2.229–4.926, *P* < 0.0001), appeared to be significant prognostic factors statistically (Table 3). Moreover, the7-microRNA signature risk score model has a significant association with survival as exhibited by multivariate COX regression coefficients by justifying other clinical factors (HR = 1.091, 95% CI 1.40–4.18, *P* < 0.0001). The two other clinical factors, age (HR = 1.047, 95% CI 1.03–1.063, *P* < 0.0001) and tumor grade (HR = 2.48, 95% CI 1.636–3.76, *P* < 0.001), were found out to be independent prognosis factor. However, gender (HR = 1.187, 95% CI 0.821–1.717, *P* = 0.361) was a variable or dependent prognostic factor.

The article "Identification and Potential Mechanisms of a 7-MicroRNA Signature That Predicts Prognosis in Patients with Lower-Grade Glioma" was retracted in 2023. Reasons: signs of a paper mill; compromised peer review; unreliable results or conclusions.

### 3.4. Construction of Target Gene PPI

The targeted genomes of the seven prognostic microRNAs were identified by using TargetScan, miRTarBase, and miRDB databases. Overall, 582 gene pairs of microRNA-target were extracted and utilized for microRNA-target gene network construction (Figure 4). The STRING database and Cytoscape software were used for the construction of PPI networks. The top 20 genes, thus, determined are shown in Figure 5.

### 3.5. GO and KEGG Analyses

For verification of 7-microRNA interrelated pathways and their potential functions, GO and KEGG analyses were conducted. The investigations proved that targeted genes have various enriched GO functions, e.g., “axon development” and “axonogenesis” in the BP,“ion channel activity” and “channel activity” in the MF, and “postsynapse” and “presynapse” in the CC categories (Figure 6). KEGG analysis exhibited for those genes also were developed in tumor-associated pathways such as the “cAMP signaling pathway,” “calcium signaling pathway,” and “Wnt signaling pathway” (Figure 7).

### 3.6. Assessment of the Risk Score and Expression of Prognostic microRNAs in Different Grades of Glioma

By using TCGA, we accessed the risk score level and expression of the 7-microRNAs in glioma of grade II and grade III. Results indicated that the grade-III glioma gets higher risk score to compare with grade-II glioma (Figure 8). Risky microRNAs (hsa-miR-92b-5p and hsa-miR-221-3p) were markedly upregulated in grade-III glioma (Figure 9). Protective microRNAs (hsa-miR-3200-3p, hsa-miR-548b-3p, and hsa-miR-153-5p) were markedly downregulated in grade-III glioma. hsa-miR-221-3p showed an upregulated trend, while hsa-miR-181a-2-3p showed a downregulated trend though not statistically significant, suggesting that they could be used for screening of glioma as the potential prognosis biomarkers.

## 4. Discussion

Glioma is known for its highly infiltrative growth characteristic as the major abundant type of central nervous system tumors [4]. Previous prediction of prognosis and selection of treatment mainly depended on histology combined with IDH and 1p/19 g status examination [21, 22]. New molecular features for the prognosis and treatment of LGG raised widespread attention with the development of sequencing technology [23]. Identification of novel prognostic biomarkers as well as therapeutic agents can play a crucial role in its treatment. MicroRNAs are small RNAs with about 20 nucleotides that could activate the downstream signaling mechanism and targeted genes. Now, over 5,000 microRNAs have been found in humans, many of which have been found to have a critical function in cancer progression [24, 25]. The microRNAs can be easily detected in a variety of body fluids [26]. The stability and functionality of microRNA indicated that they may be used as prognostic markers, although the selection of the most effective diagnostic or therapeutic agent for glioma disease is a challenging process.

The article "Identification and Potential Mechanisms of a 7-MicroRNA Signature That Predicts Prognosis in Patients with Lower-Grade Glioma" was retracted in 2023. Reasons: signs of a paper mill; compromised peer review; unreliable results or conclusions.

In our study, we utilized bioinformatics approaches for the prognosis of LGG by identifying a risk model of microRNAs. A 7-microRNA prognostic model composed of the weighted expressions of hsa-miR-181a-2-3p, hsa-miR-3200-3p, hsa-miR-92b-5p, hsa-miR-10b-5p, hsa-miR-221-3p, hsa-miR-548b-3p, and hsa-miR-153-5p was successfully established. Among the seven microRNAs, 3 microRNAs were risky and 4 microRNAs were protective. Based on the model, there are two basic categories of LGG patients including the high-risk and low-risk group. The substantial variations were observed in OS among groups of low risk and high risk in the testing, training, and complete cohorts. Multivariate Cox regression represented that the 7-microRNA model could be utilized as a variable diagnostic factor within other traditional clinical parameters. We observed that the expression level of risk score was relatively lower in grade II as compared to grade III of glioma disease. Except for hsa-miR-181a-2-3p and hsa-miR-221-3p, all microRNAs exhibited notable distinguishing features among-II and grade-III glioma. To find associated genes and pathways, we applied analysis that included the coexpression network, PPI network, GO term enrichment, and KEGG pathway.

Based on the result of coexpression genes, we screened 20 hub genes from the targeted genes which might be the key therapeutic targets involved in glioma development. GO enrichment analysis concluded that “axon development” and “axonogenesis” were the most significant enrichments in the category of BP, “postsynapse” and “presynapse” in the category of CC, and “ion channel activity” and “channel activity” in the MF category. Coincidentally, Zeng et al. found the invasiveness of glioma could be prompted by the development of pseudotripartite synapses among glioma cells and glutamatergic neurons [27]. The network of neuroglial synapses produces postsynaptic ion currents that mediate the progression of gliomas [28]. Researchers have explained the main KEGG pathway results in our studies were closely related to glioma development. As considerations, Oh et al. investigated that stimulations of the cAMP signaling mechanisms involved for the cerebral conversion of glioma [29]. Activating the cAMP signaling pathway could inhibit glioma cell invasion as well as proliferation and promote apoptosis [30]. The calcium signaling pathway was screened as a pathway possibly associated with glioma cell invasion and metastasis [31]. The Wnt signaling pathway was involved in proliferation, migration, differentiation, and apoptosis [32]. Moreover, our KEGG pathway analysis also identified the association of glutamatergic synapse with glioma which has been described above. This result revealed that the tumor-promote effect of the Wnt signaling pathway may also reflect the ability to develop dendrites, axons, and synapses [33].

The article "Identification and Potential Mechanisms of a 7-MicroRNA Signature That Predicts Prognosis in Patients with Lower-Grade Glioma" was retracted in 2023. Reasons: signs of a paper mill; compromised peer review; unreliable results or conclusions.

Through our analysis, we proposed that hsa-miR-92b-5p, hsa-miR-10b-5p, and hsa-miR-153-5p may lower the survival rate of LGG patients due to destroying the cancer suppressor gene regulatory mechanism, while hsa-miR-181a-2-3p, hsa-miR-3200-3p, hsa-miR-548ba, and hsa-miR-153-5p may enhance the survival rate of LGG patients by negatively regulating LGG oncogenes. The expression of prognostic microRNAs indicated that the 7-microRNAs were associated with LGG malignant phenotype in grade-II and grade-III glioma. We also searched relative examinations to explain the roles of the 7-microRNAs in the Pubmed database. Consistent with our study, hsa-miR-181a-3p and hsa-miR-153-5p have already been verified to be expressed lower in human LGG tissue than in normal tissue and act as protective factors [34, 35]. hsa-miR-181a-3p can directly downregulate ZBTB33 expression; therefore, it inhibits the expansion, growth, invasions, and unspecialized epithelial transition of glioma tumor cells [34]. Meanwhile, antiglioma cells were possibly induced by hsa-miR-153-5p as downregulating Rictor [35]. Furthermore, hsa-miR-92b-5p, hsa-miR-10b-5p, and hsa-miR-221-3p have already been verified to be expressed higher in human LGG tissue than normal tissue and act as risk factors [36–38]. Li et al. identified that hsa-miR-92b-5p promotes glioma proliferation by promoting DKK3 and then activating the Wnt/beta-catenin signaling pathway [32]. Moreover, the downregulation of hsa-miR-10b-5p repressed spread, movement, and invasion of glioma cell by the activation of TGF-*β*1 stimulation [31] or homeobox B3 (HOXB3) expression [39]. For hsa-miR-221-3p, researchers discovered the overexpression could activate the Akt pathway [40]. Though there are few studies analyzing the expression and function of the hsa-miR-3200-3p and hsa-miR-548b-3p in LGG, the hsa-miR-3200-3p and hsa-miR-548b-3p have been reported to inhibit growth, migration, and invasion of tumor cells of the gastrointestinal tract and hepatocellular carcinoma cells separately [41, 42]. But, we still need to figure out how the hsa-miR-3200-3p and hsa-miR-548b-3p work in LGG.

The article "Identification and Potential Mechanisms of a 7-MicroRNA Signature That Predicts Prognosis in Patients with Lower-Grade Glioma" was retracted in 2023. Reasons: signs of a paper mill; compromised peer review; unreliable results or conclusions.

It was concluded that the microRNAs have a crucial function in the prognosis of tumor, its development, and also progression. In the current study, a risk assessment model constituting the seven differently expressed microRNAs has been provided, which would be helpful in the prognosis of glioma. However, a more diverse study based on several databases is required as the recent study involves the expression data of microRNA from one database only.

## Figures and Tables

**Figure 1:** (a) Significantly differentially expressed microRNAs and (b) mRNAs screened in TCGA by constructing a prognostic scoring model based on 7 prognostic microRNAs.

**Figure 2:** (a) The distribution of survival time and survival status among the two risk groups in the training, testing, and entire cohorts. The dotted line indicates the median cutoff point of the risk score that has been used for stratifying individuals with LGG into two groups of high and low risk. (b) The curves of Kaplan–Meier are dependent of the microRNA-based risk assessment model in the testing cohort, training cohort, and entire cohort of the low- and high-risk patients. (c) Representation of ROC line curves in the testing, entire, and training cohorts.

**Figure 3:** Kaplan–Meier curve expression by 7-microRNAs for high- and low-risk groups.

**Figure 4:** Coexpression network of the 7-microRNA signature.

**Figure 5:** Top 20 genes selected from the PPI network.

**Figure 6:** GO analytical representation target genes linked with 7-microRNAs.

**Figure 7:** KEGG analysis of novel genes related to 7-miRNAs.

**Figure 8:** The distributions of risk score among grade-III glioma and grade-II glioma.

**Figure 9:** Representations of the expression of the 7-microRNAs among glioma of grade II and grade III.

**Table 1:** Clinical features of study individuals with LGG for the training, testing, and entire cohort.

Clinical characteristic	Training cohort (*n* = 240)	Testing cohort (*n* = 237)	Entire cohort (*n* = 477)
Age (years, mean ± SD)	44 ± 12	41 ± 17	43 ± 13
Sex (female/male)	116/124	103/134	219/258
Mortality (deceased/alive)	178/62	177/60	355/122
Grade (G2/*G*3)	112/128	118/119	230/247
Overall survival time (years, mean ± SD)	2.9 ± 2.8	2.7 ± 2.4	2.8 ± 2.6

SD, standard deviation.

**Table 2:** Detailed properties of the seven microRNAs screened to build the risk assessment model.

Name	Type	Coefficient	HR	95% CI	*P* value
hsa-miR-181a-2-3p	Protective	−0.398	0.672	0.5–0.902	0.008
hsa-miR-3200-3p	Protective	−0.361	0.697	0.512–0.948	0.021
hsa-miR-92b-5p	Risky	0.328	1.389	1.06–1.818	0.017
hsa-miR-10b-5p	Risky	0.118	1.125	1.018–1.243	0.021
hsa-miR-221-3p	Risky	0.287	1.333	1.051–1.69	0.018
hsa-miR-548b-3p	Protective	−0.225	0.799	0.652–0.979	0.03
hsa-miR-153-5p	Protective	−0.321	0.725	0.543–0.969	0.03

The article "Identification and Potential Mechanisms of a 7-MicroRNA Signature That Predicts Prognosis in Patients with Lower-Grade Glioma" was retracted in 2023. Reasons: signs of a paper mill; compromised peer review; unreliable results or conclusions.

**Table 3:** COX regressions of univariate and multivariate coefficients for prognosis factor analysis of OS.

Variable	Univariate analysis			Multivariate analysis		
	HR	95% CI	*P* value	HR	95% CI	*P* value
Age	1.058	1.043–1.074	<0.001	1.047	1.03–1.063	<0.001
Gender	1.063	0.742–1.522	0.739	1.187	0.821–1.717	0.361
Grade	3.313	2.229–4.926	<0.001	2.48	1.636–3.76	<0.001
Risk score	1.135	1.109–1.162	<0.001	1.091	1.063–1.12	<0.001

## Data Availability

The data used to support the findings of this study are available from the corresponding author upon request.

## Abbreviations

LGG: Lower-grade glioma
PPI: Protein-protein interaction
AUC: The area under the curve
BP: Biological process
TCGA: The Cancer Genome Atlas
FDR: False discovery rate
CC: Cellular component
KEGG: Kyoto Encyclopedia of Genes and Genomes
GO: Gene Ontology
MF: Molecular function
WHO: World Health Organization
DEmicroRNAs: Differentially expressed microRNAs
ROC: Receiver operating characteristic
DEmRNAs: Differentially expressed mRNAs
OS: Overall survival
FC: Fold change.
